# Conservative Treatment and Rehabilitation Training for Rectus Femoris Tear in Basketball Training Based on Computer Vision

**DOI:** 10.1155/2022/6230025

**Published:** 2022-05-05

**Authors:** Yupeng Zhang, Gaowei Zhao

**Affiliations:** School of Physical Education, Henan Agricultural University, Zhengzhou, 450002 Henan, China

## Abstract

Computer vision is an emerging artificial intelligence subject, whose purpose is to make computers have the same ability to perceive and understand image semantic information as humans. Computer vision technology is based on high-performance computers, which can obtain massive amounts of information and data in a short period of time and use intelligent algorithms to perform high-speed data processing on the information, which is conducive to the integration of information related to product design, production process management, etc. Due to the rapid development of visual sensing technology, computer technology, and image processing technology, computer vision technology has been widely used in the fields of food, medicine, construction, chemical industry, electronics, packaging, and automobiles. This article uses computer vision technology to compare four conservative treatments and rehabilitation training for rectus femoris in basketball training and analyze the best rehabilitation treatment for rectus femoris tear. The experimental results show that the average electroacupuncture plus muscle stretching exercise group after treatment has an average EMG value of 55.49, an average muscle strength rating of five, an average motor function score of 23.45, and an average treatment recovery time of 11.6 days. This group has the best treatment effect.

## 1. Introduction

Computer vision is a new comprehensive discipline formed with the development of computer technology, which combines computer technology and engineering, signal processing, physics, applied mathematics and statistics, and other disciplines. It involves a variety of high and new technologies such as image analysis, pattern recognition, visual sensing, and signal processing. Computer vision is a subject that uses computers or corresponding devices to simulate human vision to perceive, distinguish, and recognize the physical world. It can recognize and detect objects by processing and extracting the collected image or video data. The purpose is to explore how to use computers to complete human visual functions. Compared with machine vision, which emphasizes the use of machine vision products to solve vision problems, the core of computer vision is electronic information technology, which focuses on the use of multiple information technologies to analyze vision problems. Simply put, machine vision focuses on accurate geometric calculations, while computer vision focuses on perception and recognition. At the same time, computer vision can be applied to various occasions that require visual observation. In certain dangerous, subtle, and nonvisual situations, it is significantly better than human vision.

Computer vision was developed in the 1950s. At that time, the research field was mainly focused on the analysis and recognition of two-dimensional images, including optical character recognition and microscopic image analysis. In the 1960s, people used computer programs to represent a combination of points, lines, and surfaces as objects to be recognized. Three-dimensional vision can be presented with two-dimensional images and thus began the study of computer vision in three-dimensional scenes. MIT's Artificial Intelligence Laboratory integrated research results in psychophysics, image processing, clinical psychiatry, and neurophysiology in the 1970s, constructing three completely different computer vision system frameworks, laying the foundation for computer vision. In the 1980s and 1990s, with the rapid development of artificial intelligence technology, computer vision technology became increasingly mature, and technologies such as stereo vision and stereo matching also developed rapidly and were widely used in the industrial field. In the twenty-first century, many new development directions have appeared in computer vision technology. Computer vision is deeply integrated with visual sensing technology, computer technology, and image processing technology and has various applications in transportation, security, medical treatment, and robotics.

Leg muscle strain is a common sport injury in basketball training, and its incidence is high. Leg muscle strain refers to the slight damage or partial tear of the muscle caused by active or passive overstretching of the muscle. Leg muscle strains mainly occur in the back muscles of the thigh, rectus femoris, midfemoris, adductor thigh, and gastrocnemius. Rectus femoris tears usually occur in activities such as sprinting, jumping, or kicking and are especially common in basketball training. Insufficient warm-up activities, excessive fatigue, training with injuries, or high-intensity exercise close to the game are more likely to cause strain. Once the rectus femoris tear occurs, it often affects the athlete's stepping, leg swing, and back kick technique, affecting normal training and competition, and even affecting normal life ability. At present, the commonly used treatment and rehabilitation planning methods for rectus femoris include acupuncture, external application of Chinese medicine, massage, sports, massage, and strength training.

Computer vision technology is a new interdisciplinary subject that integrates multiple technologies such as image processing, image analysis, pattern recognition, and artificial intelligence. It has the characteristics of fast, real-time, economical, consistent, objective, and nondestructive testing. It has good application prospects in medical fields such as intelligent diagnosis, intelligent treatment, imaging research, big data and conventional health service management, and humanized medicine. However, in sports training and rehabilitation, the application of computer vision technology has just started, and there is still a lot of room for development. This article briefly describes the application of computer vision technology in the rehabilitation treatment of rectus femoris muscle and compares and analyzes the four rehabilitation treatment methods through experiments to provide a reference for the application of computer vision technology in the field of sports training and rehabilitation research.

## 2. Related Work

In terms of theoretical research, domestic and foreign experts and scholars have discussed the application and development prospects of computer vision in various fields and have done relevant research on the technical aspects and applications of computer vision. Wldchen and Mder published 120 peer-reviewed studies through comparison and analysis (2005-2015). They used computer vision technology to describe the application method of the researched plant organ classification, as well as the characteristics of the plant, that is, the shape, texture, color, edge, and vein structure. They used digital cameras and mobile devices, remote access to databases, image processing, and pattern recognition technologies to achieve automated species recognition [1]. To solve the problem of centralized processing of millions of large-scale data in medical imaging in computer vision, Barbu et al. proposed a novel and efficient data processing scheme. This scheme judges constrained variables by gradually removing variables, uses one-dimensional piecewise linear response functions to explain nonlinearity, and applies second-order priors to these functions to avoid overfitting. Experiments show that the method he proposed is more accurate and quicker than other methods in regression analysis and data classification, and at the same time, it is very efficient and scalable in the algorithm [2]. Cha et al. propose a damage detection method by integrating nonlinear recursive filters and computer vision algorithms to measure the dynamic response of structures. They use motion amplification technology and optical flow algorithms to measure structural displacement and uses an unscented Kalman filter to predict structural characteristics, such as stiffness and damping coefficient. Compared with traditional methods, this noncontact displacement measurement method does not require an intensive instrument contact process. And it will not add any systematic error that may cause measurement skew to the structure, and it can measure more signals [3]. Garcia et al. believe that computer vision can be used to detect people in the Internet of Things to improve the safety of smart cities, smart towns, and smart homes. They use computer vision to analyze pictures to detect and analyze the characters in the pictures, process the pictures with sensors with two different states, and test the computer vision module in the real environment to verify its feasibility [4]. Rosa et al. applied computer vision to food certification and quality assessment in the food industry and developed a data fusion strategy. They combined the output of multiple instrument sources and used multivariate analysis to quickly and accurately assess the quality of food [5]. Decost et al. applied computer vision and machine learning methods to develop a system to characterize powdered raw materials for metal additive manufacturing (AM). It is used to create microstructure-scale image representations that can be used for clustering, comparing, and analyzing powder photomicrographs. When using eight kinds of commercial raw material powders, the system classifies the powder images into the correct material system with an accuracy rate of over 95%. The results show that objective powder raw material standards can be defined based on visual images [6]. Dong et al. integrate computer technology into tea research. They believe that human sensory evaluation is easily affected by many factors such as light, experience, psychology, and vision. At the same time, people may distinguish subtle differences between similar colors or textures, but it is difficult to determine the specific content of the tea. Because the description of color and texture by human beings is qualitative, it is difficult to accurately, standardly, and objectively evaluate the sensory quality. The author uses computer vision image technology to establish a quantitative evaluation model of tea quality and make a quantitative evaluation of tea quality [7].

## 3. Computer Vision and Convolutional Neural Networks

### 3.1. Computer Vision

Computer vision is to analyze and calculate the symbols and numbers of images and videos to realize the recognition, detection, and tracking of targets. Computer vision tasks mainly include four aspects, namely, image recognition, target detection, image segmentation, and target tracking. It is shown in Figure 1. Image recognition is the most basic work in a computer vision system, and its purpose is to recognize the object information in the image. At present, there are two main types of image recognition technologies, one is based on traditional machine learning algorithms, and the other is various types of recognition networks based on deep learning. In practical applications, image recognition is mainly for the recognition of specific targets [8], for example, license plate recognition. At the ETC entrance of the expressway, there is no manual toll, and the camera can recognize the license plate and charge the corresponding fee. In addition, face recognition has also been widely used in daily life, such as Alipay's face payment system. Target detection is based on the recognition of the target through the computer to locate the object in the image and determine its classification. One of the commonly used target detection methods is to detect pedestrians. At intersections, pedestrians under surveillance can be quickly detected, the number of pedestrians can be estimated, and abnormal conditions can be warned. Image segmentation is a method for the computer to interpret images. On this basis, a semantic-based image segmentation method has emerged. Image semantic segmentation is to divide the image into different objects and classify them and then understand the meaning of each pixel in the image from the semantic level. It combines semantic segmentation of the image with target detection, segmenting the image into individual objects, and outputting them with the position of each object. Target tracking refers to tracking one or more objects to be noticed in a specific environment, to separate the tracked object from the background and track it. In UAV and video surveillance, target tracking is currently a widely used method [9].

Figure 2 shows the distribution of the computer vision industry chain. The computer vision industry chain is divided into three parts: the basic layer, the technical layer, and the application layer. The basic layer is the foundation of the computer vision industry chain, providing massive data and a variety of different algorithm support for the computer vision system. It mainly includes two parts: core hardware and basic algorithm. In addition to the chip, the core hardware also has a vision sensor with image processing functions. The chip is the most basic algorithm foundation, including GPU, CPU, FPGA, and ASIC. Among them, the self-defined image processing chip can provide better image processing performance while consuming very little energy. Basic algorithm vendors provide basic models and frameworks for computer vision technology, including R-CNN, Fast-RCNN, Faster-RCNN, and YOLO [10, 11]. In the computer vision industry chain, the technical layer is a key link. It provides enterprises with computer vision technical support so that they can adapt to the application requirements of various industries and various scenarios. Technical research focuses on computer vision tasks, including image classification, target detection, image semantic segmentation, and target tracking [12]. The application layer is an extension of the computer vision industry. It meets the requirements of specific application scenarios through a combination of software and hardware. The application layer includes two parts: system solutions and final product development. The application range of computer vision is very broad. It can be used in applications such as smart security, face recognition, ADAS, vision solutions and can also be integrated into a series of final products such as drones, robots, and unmanned vehicles.

According to the data compiled by the China Academy of Information and Communications Technology, as shown in Table 1, the artificial intelligence market has increased from 11.24 billion yuan in 2015 to 55.4 billion yuan in 2019, and the artificial intelligence industry is developing rapidly.  Figure 3 shows the investment and financing situation of the artificial intelligence industry in 2019. It can be seen that the two major areas with the most artificial intelligence investment and financing events are platform applications and computer vision technology, accounting for 36.8% and 36.5%, respectively; voice technology accounted for 11.4%, and basic algorithms and chip processing accounted for 8.39% and 6.91%, respectively. On the whole, computer vision and platform applications are the most attractive areas for investment in the artificial intelligence industry.

### 3.2. Convolutional Neural Network

In many fields such as computer vision, speech recognition, and natural language processing, artificial intelligence has made remarkable achievements in various aspects. Currently, convolutional neural networks are the most commonly used method among various deep learning models. It has broad application prospects in image classification, target detection, face recognition, pedestrian recognition, and other fields [13]. The convolutional neural network is a multilevel neural network, which includes the feature information of the convolutional layer and the sampling layer. It abstracts the original data from one level through a series of operations such as convolution, pooling, and nonlinear activation function mapping. On this basis, the corresponding characteristic function is drawn and transformed into the function value of the specific task objective. A typical convolutional neural network includes an input layer, a convolutional layer, a downsampling layer (i.e., a pooling layer), a fully connected layer, and an output layer, as shown in Figure 4. In a convolutional neural network, from input to output, different computational neural nodes are used to transmit the input information level by level. It uses continuous convolution pooling technology to decode, deduce, and converge feature signals, map them to the hidden layer feature space, and classify them for output [14, 15].

#### 3.2.1. Convolution Operation

Convolution is an important analysis operation in mathematics, and it is a mathematical operator. It is the third function composed of two functions *f* and *g*. This function is characterized by the overlapping area of the functions of *f* and *g* through inversion or translation [16]. The calculation formula is generally expressed by the following formula:

(1) $$\begin{array}{c} z\left(t\right)≝f\left(t\right)*\text{g}\left(t\right)=\overset{\infty }{\underset{\tau =-\infty }{\sum }}f\left(\tau \right)\text{g}\left(t-\tau \right). \end{array}$$

The integral form is:

(2) $$\begin{array}{c} z\left(t\right)=f\left(t\right)*\text{g}\left(t\right)=\int_{-\infty }^{\infty }f\left(\tau \right)\text{g}\left(t-\tau \right)d\tau =\int_{-\infty }^{\infty }f\left(t-\tau \right)\text{g}\left(\tau \right)d\tau . \end{array}$$

In image processing, an image can be seen as a two-dimensional discrete function composed of *f* (*x*, *y*) [17]. It assumes that there is a two-dimensional convolution function *g* (*x*, *y*), and the output image *z* (*x*, *y*) can be expressed by the following formula:

(3) $$\begin{array}{c} z\left(x,y\right)=f\left(x,y\right)*g\left(x,y\right). \end{array}$$

This formula can be used to extract image features when inputting a two-dimensional image. In deep learning applications, the input is a color image containing RGB three channels. The image is composed of each pixel, then such input is a high-dimensional array of 3∗image width∗image length. The corresponding convolution operation is expressed as follows:

(4) $$\begin{array}{c} z\left(x,y\right)=f\left(x,y\right)*g\left(x,y\right)\underset{t}{\sum }\underset{h}{\sum }f\left(t,h\right)g\left(x-t,y-h\right). \end{array}$$

The integral form is:

(5) $$\begin{array}{c} z\left(x,y\right)=\left(f*g\right)\left(x,y\right)=\iint f\left(t,h\right)g\left(x-t,y-h\right)dtdh. \end{array}$$

If a convolution kernel of size *m*∗*n* is given, there are:

Among them, *f* represents the input image, *g* represents the convolution kernel, and *m* and *n* are the sizes of the kernel.

Commonly used nonlinear activation functions include Sigmoid function, tanh function, ReLU, and ELU function [18, 19], and the forms are as follows:

(6) $$\begin{array}{c} \text{sigmoid}\left(x\right)=\frac{1}{1+e^{-x}}, \end{array}$$

(7) $$\begin{array}{c} \tanh\left(x\right)=\frac{e^{x}-e^{-x}}{e^{x}+e^{-x}}, \end{array}$$

(8) $$\begin{array}{c} y\left(x\right)=\left\{\begin{array}{c} x,x\geq 0,\\ 0,x<0, \end{array}\right. \end{array}$$

(9) $$\begin{array}{c} f\left(x\right)=\left\{\begin{array}{c} x,x>0,\\ \alpha \left(e^{x}-1\right),x\leq 0. \end{array}\right. \end{array}$$

#### 3.2.2. Convolutional Layer

In the convolutional layer, one or more convolution kernels (also called filters), the convolution operation is used to extract pixel-level image features, and the result of the convolution operation is transformed by the activation function mapping to form a characteristic mapping relationship from input to output. Each convolution kernel uses a sliding window to scan each feature, through the fusion of each feature information, to complete the description of the local features of the image [20].

Taking a two-dimensional image as an example, formula (6) can be transformed for the convenience of calculation, and the form of the convolutional layer becomes:

(10) $$\begin{array}{c} z\left(x,y\right)=f\left(x,y\right)*g\left(x,y\right)=m\underset{n}{\sum }f\left(x-m,y-n\right)g\left(m,n\right). \end{array}$$

Among them, *f*represents the input, which is generally a two-dimensional image, *g* represents the convolution kernel, and *m* and *n* represent the sizes of the convolution kernel. To express more intuitively, Algorithm 1 shows the working process of the convolutional layer.

Among them, input: feature map Input, width Width1, length Height1, and depth Depth1.

Hyperparameters: convolution kernel size *F*, step Stride, number of convolution kernel *K*, and fill factor *P*.

Output: feature map Output after convolution, width Width2, length Height2, and depth Depth2.

#### 3.2.3. Pooling Layer

Normally, a convolutional neural network will periodically insert a pooling layer into an adjacent convolutional layer. According to the perception that the beneficial image characteristics of one area are likely to be the same in other areas, the pooling layer combines semantically similar features and uses pooling operations to reduce the feature vector output by the convolutional layer, while avoiding overfitting [21]. In the feature map, the pooling unit can calculate the local block value. Adjacent pooling elements can be read once in a small area, thereby reducing the dimension of data expression. This ensures that the translation of the data remains unchanged, thereby greatly reducing the number of parameters and the amount of calculation [22]. The processing process of the pooling layer is similar to that of the convolutional layer. As shown in Algorithm 2, only the depth of the feature map after pooling and the depth before pooling are not changed.

In the pooling layer, *F* represents the size of the pooling unit, and other parameters are the same as the convolutional layer.

Maximum pooling (MaxPooling), average pooling (MeanPooling), and random pooling methods are currently the most common pooling methods, as shown in Figure 5.

Different pooling methods have different pooling results. The maximum pooling operation uses the maximum value of the image area as the result of the pooling of this area; while the average pooling method calculates the average value of the image area, the final value of the random pooling algorithm is randomly selected according to the size of the probability matrix. The three pooling methods in Figure 5 all use a filter with a size of 2∗2. The step is 2, traversing the entire input, and the result obtained is 1/4 of the original size. After the pooling operation, 75% of the result value is discarded, which saves the computational cost of the network.

#### 3.2.4. Fully Connected Layer

The fully connected layer is located in the previous layer of the output of the convolutional neural network structure and has a multilayer perception function, as shown in Figure 6. The neurons of each fully connected layer are completely connected to the neurons of the previous layer, and the name of the fully connected layer comes from this [23]. The final output of the network is the high-level features of the input image, and the classification algorithm is used to calculate the corresponding classification results. The Softmax regression classification model [24] is usually the final level of the fully connected level, and the result is the value in each category between 0 and 1.

In a computer, a fully connected layer is equivalent to a network structure formed by inner product operations between neural nodes, including forward and reverse operations [25]. The forward operation uses formula (11) to calculate the output value of each neuron, and the reverse operation uses formula (12) to calculate the error term of each neuron.

(11) $$\begin{array}{c} y=W^{T}x+b, \end{array}$$

(12) $$\begin{array}{c} \frac{\partial l}{\partial x}=W*\frac{\partial l}{\partial y},\frac{\partial l}{\partial w}=W*{\left(\frac{\partial l}{\partial y}\right)}^{\text{T}}. \end{array}$$

Among them, *y* ∈ *R*^*m*×1^ represents the output of the neuron, x∈R^n×1^ represents the input of the neuron, *W* ∈ *R*^*n*×*m*^ represents the weight of the neuron, *b* is the bias term, and *l* is the neuron of the layer.

The reverse transmission process combines two forms of reverse propagation and algorithm optimization. It uses the optimal algorithm to correct the error signal and fine-tune the network model. It calculates the gradient of each loss function in the network and then feeds it back to the optimal algorithm, so that it can get the smallest loss function or cost function [26]. That is to say, in the back propagation, the chain rule is used to perform iterative operations on each neuron node, to compare the actual output with the corresponding expected output. Assuming that the loss function is determined in the form of a square error function, the loss function can be expressed as follows:

(13) $$\begin{array}{c} E^{n}=\frac{1}{2}\overset{c}{\underset{k=1}{\sum }}{\left(t_{k}^{n}-y_{k}^{n}\right)}^{2}=\frac{1}{2}{\left\|t^{n}-y^{n}\right\|}^{2}. \end{array}$$

This formula represents the training error of the data sample *n*, *c* represents the number of nodes in the output layer, generally the number of the final classification, *t* represents the appropriate training sample size, and *y* represents the output of the network training. To minimize the error, it is usually necessary to modify the weight matrix, and its adjustment direction can be expressed by the following formula:

(14) $$\begin{array}{c} ∆W^{l}=-\eta \frac{\partial E}{\partial W^{l}},\\ \frac{\partial E}{\partial W^{l}}=x^{l-1}{\left(\delta^{l}\right)}^{T},\\ \delta =\frac{\partial E}{\partial b}=\frac{\partial E}{\partial u}∙\frac{\partial u}{\partial b}. \end{array}$$

The corresponding residual of the middle layer of the convolutional network is:

(15) $$\begin{array}{c} \delta^{l}={\left(W^{l+1}\right)}^{T}⊙f\left(u^{l}\right). \end{array}$$

Correspondingly, the residual of the last layer *L* of the network is:

(16) $$\begin{array}{c} \delta^{L}=f\left(u^{l}\right)⊙\left(y^{n}-t^{n}\right). \end{array}$$

Since the convolutional neural network contains different levels, formula (15) is generally converted into the following formula to find the residual error in the convolutional neural network:

(17) $$\begin{array}{c} \delta^{l}={\left(W^{l+1}\right)}^{T}\delta^{l+1}⊙f\left(u^{l}\right). \end{array}$$

In summary, the backpropagation algorithm starts from the last layer, performs reverse operations on the error vector, and uses the chain law repeatedly. It calculates the loss of the cumulative gradient through the inverse operation, to minimize the loss function. In this way, in the convolutional neural network, the backpropagation training method can be described as the training algorithm in Algorithm 3.

Among them, the input value is the loss function *E*; the output value is the gradient of the loss function.

## 4. Experimental Design

From March 2021 to October 2021, 48 patients with mild strains of the posterior thigh muscles were selected from the Tuina, Rehabilitation and Acupuncture Departments and wards of the First Affiliated Hospital of Nanchang University and the Second Affiliated Hospital of Nanchang University. All cases were examined by imaging DR and MRI, and the judging standard was tested by sports medicine or modern medicine. The manifestation was a muscle strain caused by a slight rectus femoris tear or a closed injury caused by a slight tear. They were numbered according to the time of visit and were randomly divided into four groups. They were Chinese medicine + massage group (12 cases), acupuncture + moxibustion treatment group (12 cases), electroacupuncture plus muscle stretching exercise group (12 cases), and control group (12 cases). The average rectus femoris myoelectric value (AEMG), rectus femoris muscle strength test, MMT, lower limb motor function, and rehabilitation time were compared between the four groups before and after treatment.

Group 1: the traditional Chinese medicine + Tuina massage group first used saffron and Panax notoginseng soaked medicinal wine for external application and massage to experiment and intervene the patients, using rubbing, kneading, pressing, and other techniques to promote the absorption of medicinal effects and basic massage for 10 minutes. Rehabilitation treatment was carried out by massage method, pressing each acupoint on the thigh for 10 minutes to prepare for massage. Then, use fingers, palms, elbows, and other parts to apply pressure, from light to heavy, from shallow to deep, and press on the injured rectus femoris or acupuncture points in turn. When it reaches a certain level, pause for 10-30 seconds, then slowly relax and repeat several times.

Group 2: acupuncture + moxibustion treatment group selects the injured muscles to be disinfected with alcohol first. At both ends and sides of the abdominal muscles after injury, choose milli needles according to the depth of the injured muscle, and use needles about 1 to 2 inches along the painful area. After that, the patients in this group were treated with moxibustion for rehabilitation. The moxibustion box was fixed on the injured part of the thigh, and the heat was as high as the patient could bear for 30 minutes.

Group 3: the electrical acupuncture and muscle stretching training group performed routine disinfection on the injured thigh of the patient. According to the depth of the injured muscle, acupuncture needles were used to puncture the painful area, 1 to 2 inches away from the painful area. After acupuncture, one time, add the electrode, the painful part is in contact with the negative electrode, and the density wave is selected, the frequency is 60-100 times/min, the intensity is within the tolerance of the patient, and it lasts for 20 minutes. After the electroacupuncture therapy, stretch the leg muscles several times a day, stretch for 30-60 seconds each time, and repeat it many times. When stretching exercises, be gentle and have a certain muscle stretching feeling, but do not let the wound have severe pain.

Group 4: the control group adopts physical therapy of rest and ice compress, and the daily activities, diet, work, and rest requirements are as consistent as possible with other experimental groups.

### 4.1. Average Rectus Femoris Myoelectric Value AEMG

The patient lies flat and routinely disinfects the injured part of the thigh, fixes the electrode sheet on the abdomen of the rectus femoris, allows the patient to perform flexion and extension exercises, and measures the average electromyographic value of the rectus femoris with an electromyography meter. The abscissa of Figure 7 is different between test samples, each group has 12 cases, and the ordinate is the average electromyographic value of the rectus femoris muscle. The average EMG value of the rectus femoris muscle before treatment in group 1 was 39.44, and the average EMG value after treatment was 55.49. The average EMG value of the rectus femoris muscle before treatment in group 2 was 39.03, and the average EMG value after treatment was 59.59. The average EMG value of the rectus femoris muscle before treatment in group 3 was 37.71, and the average EMG value after treatment was 62.08. The average EMG value of the rectus femoris muscle of the control group 4 before treatment was 39.47, and the average EMG value after treatment was 44.46. It can be seen from Figure 7 that the average rectus femoris myoelectric value after treatment was significantly higher than that before treatment. Among them, group 3 had the largest change in the rectus femoris myoelectric value before and after treatment, and the treatment effect was the best.

### 4.2. Rectus Femoris Muscle Strength Examination, MMT

The abscissa is different between test samples, each group has 12 cases, and the ordinate is the MMT muscle strength assessment grade. The first level is that the muscles are slightly contracted, but the joints cannot be moved, and the muscle strength is 10% of the normal muscle strength. The second level is that muscle contraction can make the limbs perform a full range of joint activities under the condition of removing gravity, and the muscle strength is 25% of the normal muscle strength. The third level is that the muscle contraction can make the limbs resist gravity to do the full range of joint activity, but cannot resist the external resistance, and the muscle strength is 50% of the normal muscle strength. The fourth level is that muscle contraction can make the limbs resist gravity and some external resistance, and the muscle strength is 75% of the normal muscle strength. The fifth level is that muscle contraction can make the limbs resist gravity and fully resist external resistance, and the muscle strength is 100% of the normal muscle strength. In group 1, the average muscle strength of the rectus femoris before treatment was grade 3, and the average muscle strength after treatment was grade 4. In group 2, the average muscle strength of the rectus femoris before treatment was grade three, and the average muscle strength after treatment was grade four. In group 3, the average muscle strength of the rectus femoris before treatment was grade 4, and the average muscle strength after treatment was grade 5. It can be seen from Figure 8 that the MMT classification of the three groups after treatment was significantly improved compared with that before treatment, and the rectus femoris muscle strength evaluation classification of group 3 was the best after treatment, and the muscle strength of the muscle group was the best.

### 4.3. FMA Score of Lower Limb Motor Function

The Fugl-Meyer motor function score was used to evaluate the ability of the lower limbs to complete exercise. The maximum score is 34 points, a total of 17 inspection items, and the highest score is 2 points. The higher the score, the better the lower limb mobility. In group 1, the average score of lower limb motor function before treatment was 10.81, and the average score of motor function after treatment was 17.18. In group 2, the average score of lower limb motor function before treatment was 10.87, and the average score of motor function after treatment was 21.92. In group 3, the average score of lower limb motor function before treatment was 10.59, and the average score of motor function after treatment was 23.45. It can be seen from Figure 9 that the FMA scores of lower extremity motor function of the three groups of patients were significantly improved than before treatment. Among them, group 3 had the highest FMA score and the best lower extremity motor function.

### 4.4. Recovery Time

The horizontal and vertical coordinates are the test samples of each group and the recovery time of the corresponding patients. The average treatment recovery time of group 1 was 16.8 days, the average treatment recovery time of group 2 was 14.6 days, the average treatment recovery time of group 3 was 11.6 days, and the average treatment recovery time of group 4 was 26.8 days. It can be seen from Figure 10 that the average treatment recovery time of group 3 is the shortest, and the recovery speed of the injured part of the patient is the fastest. The recovery time of group 2 is also shorter, and the treatment effect is faster.

## 5. Discussion

Rectus femoris tear refers to the fact that the rectus femoris muscle is affected by an external forces, causing muscle fiber breakage and capillary rupture, that is, the front rectus femoris muscle of the thigh is torn. The pathological changes include local hemorrhage, edema, cell degeneration, pain, restricted mobility, hardening, and thickening of muscle fibers. Traditional Chinese medicine + Tuina massage is easy to operate and has a wide range of applications in the rehabilitation of rectus femoris tears. Compared with the control group, traditional Chinese medicine treatment has an obvious effect in the rehabilitation of rectus femoris tear, but it is far inferior to acupuncture + moxibustion treatment and electric acupuncture combined with muscle stretching exercises. Among the rehabilitation treatment methods used in the experiment, the effect of electroacupuncture combined with muscle stretching exercises is the most obvious. The rectus femoris myoelectric value changes the most, and the treatment effect is the best; the muscle strength rating is the best, and the muscle strength is the best. The FMA score is the highest and the lower limb motor function is the best; the average treatment recovery time is the shortest, and the recovery efficiency is the highest. Electroacupuncture treatment of rectus femoris muscle can relieve muscle and blood, relieve pain, promote local blood circulation, eliminate inflammation and edema, regulate nerve excitability, relax muscle adhesions, and reduce muscle spasms. In the process of treating the rectus femoris muscle, muscle stretching also plays an important role. It can promote muscle circulation, reduce muscle cramps, and avoid muscle contractures and adhesions caused by injury. This is an important training for improving the quality of muscle recovery, preventing muscle strain, and helping to break through contraction training.

The traditional Chinese medicine treatment method is to use Chinese medicine and Tuina massage. However, due to the long treatment period, it takes some time for the recovery of motor function, which will greatly affect the continuity of training and even lead to serious consequences. After injury, muscle fibers proliferate and form inflammatory adhesions, inflammatory tissue contracture, degeneration, and loss of elasticity, resulting in cord-like changes, resulting in changes in the original structure and composition, and resulting in loss of muscle function. The symptoms are constant pain, easy to tear again, and can affect the surrounding joints. Electroacupuncture combined with muscle stretching exercises combines electroacupuncture treatment and muscle stretching exercises to avoid local stimulation, facilitates the elimination of muscle inflammation, improves blood circulation in the injured area in time, effectively prevents muscle adhesion and spasm, and quickly restores damage. Therefore, electroacupuncture combined with muscle stretching exercises has the characteristics of good curative effect, short course of treatment, and less sequelae. It meets the high requirements for treatment after rectus femoris tear and is worthy of promotion and further research and discussion.

## 6. Conclusion

With the extensive research and application of computer vision technology in the medical field, various image analysis technologies are used in clinical treatment of medicine. This article is based on computer vision technology, through imaging, DR, and MRI examination, for the rehabilitation of rectus femoris tear. It compares traditional Chinese medicine + massage, acupuncture + moxibustion, electric acupuncture with muscle stretching exercises, and physical therapy of rest and ice, and it analyzes the average rectus femoris myoelectric value, rectus femoris muscle strength test, lower limb motor function FMA score, and recovery time of the four therapies. Studies have confirmed that electric acupuncture combined with muscle stretching training can improve the muscle spindle function of the rectus femoris and enhance the control function of the femoral nerve to the rectus femoris, thereby significantly restoring the rectus femoris sensory and motor abilities. Compared with the other three rehabilitation treatment methods, electroacupuncture combined with muscle stretching exercises has a better therapeutic effect. Of course, there are still some shortcomings in the research of this article. The sample size selected in the experiment is too small, only 48 cases of muscle injury patients are selected, each group has only 12 cases, the sample size can be increased, and the conclusions drawn in this way are more convincing. At the same time, the time span can be larger and can be extended to a whole year.

## Figures and Tables

**Figure 1:** The main tasks of computer vision.

**Figure 2:** Computer vision industry chain.

**Figure 3:** The investment and financing segments of the artificial intelligence industry in 2019.

**Figure 4:** Convolutional neural network structure diagram.

**Figure 5:** Common pooling methods.

**Figure 6:** Fully connected layer network structure.

**Figure 7:** Changes of myoelectric value of rectus femoris before and after treatment. (a) The average electromyographic value of the rectus femoris before treatment in each group. (b) The average myoelectric value of the rectus femoris muscle after treatment in each group.

**Figure 8:** MMT classification before and after treatment. (a) The MMT muscle strength assessment grading of the rectus femoris before treatment in group 1, group 2, and group 3. (b) The MMT muscle strength assessment grading of the rectus femoris after treatment in group 1, group 2, and group 3.

**Figure 9:** Motor function of lower limbs before and after treatment. (a) The FMA score of lower limb motor function before treatment in group 1, group 2, and group 3. (b) The FMA score of lower limb motor function after treatment in group 1, group 2, and group 3.

**Figure 10:** Treatment recovery time for each group. (a) The treatment recovery time of patients in group 1 and group 2. (b) The treatment recovery time of patients in group 3 and group 4.

**Algorithm 1:** The processing flow of image features in the convolutional layer.

**Algorithm 2:** The processing flow of image features in the pooling layer.

**Algorithm 3:** 

**Table 1:** China's artificial intelligence industry market scale from 2015 to 2019.

Time	Market size/100 million yuan
2015	112.4
2016	141.9
2017	237.4
2018	415.5
2019	554

## Data Availability

The data underlying the results presented in the study are available within the manuscript.
